The article "An Evaluation Model of Career Happiness and Job Performance of Political Teachers Based on Correlation Analysis in Positive Emotional Environment" was retracted in 2023. Reasons: signs of a paper mill; suspected computer-generated content; unreliable results or conclusions; concerns about the data.

# An Evaluation Model of Career Happiness and Job Performance of Political Teachers Based on Correlation Analysis in Positive Emotional Environment

**DOI:** 10.1155/2022/2653998

**Published:** 2022-09-12

**Authors:** Ming Zheng

**Affiliations:** Chengyi University College Jimei University, Xiamen 361021, China

## Abstract

In terms of the teaching profession, the term “teacher happiness” refers to a spiritual encounter one has while practising their profession. Teachers believe that they can fulfil their needs and recognise their worth through their work in education and teaching, which will ultimately lead to happiness. Happiness is a necessary condition for teachers to perform well in the classroom, a strong foundation for professional success, the inner motivation for teachers' professional development, and the ultimate goal of education. In order to comprehend how the two affect one another, the purpose of this essay is to investigate the connection between political teachers' career satisfaction and job performance. The findings indicated that three factors, namely, work commitment, human-machine facilitation, and task performance, can also be used to categorise political teachers' career satisfaction. The overall rating of job performance and the elements affecting teachers' occupational well-being are significantly correlated. The typical *r*-correlation coefficient was 0.65. Political educators will perform better at work on a daily basis as a result of their improved occupational well-being.

## 1. Introduction

In recent years, the importance of education has become more and more obvious, and the world is paying more and more attention to education. The success of education has a lot to do with teachers. The professional responsibility of teachers is to teach and educate people. A large part of improving the quality of education revolves around teacher research. At present, most schools study the career well-being and job performance of political teachers separately and analyze their current situation and influencing factors separately. In the long run, teachers' job performance cannot be effectively improved, which affects teachers' classroom teaching quality and delays the development of the education industry. Among the existing researches, the attention on teachers' occupational well-being and job performance is relatively low. The correlation between satisfaction and job performance was explored.

The problem of teachers' occupational well-being has gradually attracted the attention of the society. In order to improve teachers' well-being, many scholars have made various related research work on it. Kim et al. investigated the influence of preservice kindergarten teachers' well-being and creative personality on their thinking styles and made a research survey. The results of the study showed that there is a correlation between well-being and creative personality, but not with the subfactors of well-being, and the influence of preservice kindergarten teachers' well-being on thinking styles can affect future goals [1]. Jung and Kim investigated the impact of preschool teachers' perceived social support on well-being and emotional intelligence, and the results showed that preschool teachers' perceived social support was in the order of information support, emotional support, evaluation support, and material support. The well-being of preschool teachers is positive and negative, and it is found that the social support perceived by preschool teachers has a significant impact on well-being in various fields [2]. Fedorov et al. analyzed the phenomenon of occupational well-being in Western and Russian psychology and sociology, defining the state of occupational activity processes and individual attitudes towards outcomes in the multivariate structure of social and psychological well-being through its fundamental determinants. To measure teachers' occupational well-being, methods of decomposition, psychometrics, mathematics, and statistical data processing were applied, and this study contributes to negatively impacting secondary school teachers' occupational well-being [3]. Skachkova and Klimenko conducted a survey study to analyse the subjective well-being indicators of scientists and educators at top Russian universities based on applied research. The study's findings demonstrated that among the university faculty members who participated in the survey, situational positive emotions outweighed negative emotions, and their level of happiness was marginally higher than the Russian population's average [4]. Several academic studies have made significant contributions to the improvement of teachers' occupational well-being, but few of these studies address the link between occupational well-being and job performance. The relationship between the two is covered in this article.

The article "An Evaluation Model of Career Happiness and Job Performance of Political Teachers Based on Correlation Analysis in Positive Emotional Environment" was retracted in 2023. Reasons: signs of a paper mill; suspected computer-generated content; unreliable results or conclusions; concerns about the data.

Workplace performance and occupational well-being are somewhat correlated. Both work performance and personal happiness are influenced by one's state of well-being. Numerous academics have studied how the two are related. Employee intrapreneurship was positively correlated with job engagement of employees with high (relatively low) sensitivity to rewards (behavioural method systems), and as a result, with creativity and innovativeness [5]. Gawke investigated how employees' reinforcement sensitivity defines the relationship between their intrapreneurial behaviour, subjective well-being, and other rated job performance. The findings highlighted the impact of acceptance on daily occupational well-being, resource savings, and motivational benefits and demonstrated that acceptance is associated with increased resilience to daily negative work events [6]. To examine the role of acceptance in the relationship between daily negative work events and occupational well-being, indicated N predicted that acceptance buffers the adverse effects of negative work events on daily well-being. Kaabomeir et al. conducted a causal comparative study to examine the impact of work-family facilitation on nurses' job satisfaction and career success, and they discovered that both work-family and home-work facilitation could predict nurses' job satisfaction and career success [7]. The relationship between developmental human resource (HR) practises and employee task performance was examined by Marescaux et al., who included well-being as a mediator along with health-related factors like exhaustion and affective organisational commitment. In light of the experimental findings, a configurational approach to human resource management, benefits, and employee performance is required, with line manager behaviour serving as a key component of the HRMS and formal HR practise [8].

In order to study the correlation between the occupational well-being of political teachers and their job performance, this paper understood the relationship between the two and selected 200 political teachers in the form of a questionnaire survey to investigate their well-being and job performance. The experimental results showed that there is a significant relationship between the total score of job performance and the four factors of teachers' occupational well-being, and the average correlation coefficient *r* reached 0.65. There is a relationship between the total score of political teachers' occupational well-being and the three factors of job performance. And there is a significant relationship, and the average correlation coefficient reached 0.73. The results showed that the job satisfaction of political teachers has a significant correlation with their job performance, and it increases with the increase of their job satisfaction.

## 2. Influencing Factors of Teachers' Well-Being

### 2.1. Teachers' Happiness

- Definition

Teachers' well-being refers to the happiness on the spiritual level obtained after the material needs are met in daily life [9]. This kind of spiritual happiness can be obtained not only from life but also from the active creation of teachers in their careers, as well as from their experience of the profession in teaching activities. It is a life state of the subject of education, and also, a life state in which teachers can freely realize their professional ideals in their own teaching activities.

(ii) Status of teachers' well-being
  1. Too much work pressure

A lot of work pressure will be placed on middle school teachers and college professors at their jobs, based on the current state of education. The first is the hours of operation. In addition to teaching, middle school teachers today also need to oversee morning and evening self-study. Teachers of the graduating class in particular need to put in more time and effort to find a solution to the enrollment rate issue. The pressure of having a professional title is the second. Today's teachers at prestigious colleges and universities must continually invest their time in raising their academic qualifications and producing scientific research findings in order to advance their professional titles. This adds to their stress levels, particularly for younger teachers who have less responsibility and lower professional titles. Teachers spend a lot of time in a bored and tense environment, which frequently results in negative emotions and has a negative impact on the person's mental health.

(2) Poor physical and mental health

The teaching profession often requires standing, talking, and sitting for a long time, which usually leads to a series of health problems, such as cervical spondylosis, back pain, and pharyngitis. At present, many teachers are already in a subhealth state, and they all have health problems more or less. The second is mental health. Students are dissatisfied with teachers' mistakes, the learning situation of the classes they bring, parents' high expectations for teachers for their children, and the promotion of their own titles, which are all psychological burdens for teachers. If these psychological burdens cannot be solved well, the accumulation may lead to the occurrence of psychological diseases.

(3) Lower overall happiness

Research surveys in recent years have found that most vocational teachers in schools are satisfied with their current jobs, but some teachers still complain about their current work status and have low occupational happiness [10]. There is a large gap in occupational happiness among different teachers, such as different genders, different regions, different ages, and different substitute subjects. Compared with primary and secondary school teachers, current college teachers are more satisfied with the quality of life than primary and secondary school teachers, and they can feel more positive emotions. Under the influence of research tools, research objects, regions, and other factors, there are obvious differences in the job well-being of university teachers in terms of gender, professional title, and teaching age. However, it is certain that the current job well-being of university teachers needs to be further improved.

(iii) Factors affecting teachers' well-being

1. Social factors

First of all, due to the lack of professional recognition of teachers in the society, their social status is low. In today's rapid development of the Internet, teachers' professional quality is often not widely recognized by the society [11]. In the eyes of many people, teachers are a profession in the middle and lower classes of society. Even teachers themselves feel that their status in society is not very high. Secondly, the society has high requirements for teachers. The current society has new requirements for teachers' teaching and teachers' professional quality. Teachers must keep pace with the times. However, older teachers will reduce their work efficiency, thus affecting the well-being of students.

(2) School factor

The management of most schools is not humane enough, which will greatly affect all aspects of teachers [12]. Due to the lack of people-oriented concept, the school only focuses on the learning situation of students and the rate of admission. However, ignoring the needs of teachers makes teaching activities more and more mechanized and rigid, thus affecting the enthusiasm of teachers. At the level of teaching methods, because the evaluation system pays too much attention to students' scores, teachers often have to adopt immutable teaching methods in pursuit of improving students' test-taking ability. However, ignoring the students' own emotional attitudes makes many students complain to teachers, making it difficult for teachers to have a high level of happiness.

(3) Personal factors

When in the same environment, some teachers can feel happy, while some teachers complain about their profession. The most important reason is internal factors. Because teachers' individual goals are not clear, many teachers' happiness is not high. When many teachers are teachers, they do not know what they want. They only want a stable salary and have no enthusiasm for the work of teachers, let alone the happiness of work.

The article "An Evaluation Model of Career Happiness and Job Performance of Political Teachers Based on Correlation Analysis in Positive Emotional Environment" was retracted in 2023. Reasons: signs of a paper mill; suspected computer-generated content; unreliable results or conclusions; concerns about the data.

### 2.2. Inner Relationship between Teachers' Well-Being and Job Performance

1. Source of job performance comes from life satisfaction

Research showed that there is an inevitable connection between teachers' work performance and their sense of well-being [13]. That is, teachers' well-being comes from work performance to a certain extent, and the quality of work performance is also affected by teachers' well-being. At the same time, job challenge is an important factor affecting job well-being and job satisfaction, and there is a significant positive relationship between job satisfaction and homework in highly challenging jobs. Job satisfaction is the main factor affecting job performance, and job satisfaction is a reflection of life satisfaction, which indicates that only teachers with a high level of life satisfaction can effectively improve their job performance.

(2) Motivation of job performance comes from emotional factors

According to studies, people who are contented are more likely to attribute their failures to outside forces [14]. They therefore recover more quickly from setbacks than people who are unhappy do, and they pursue more opportunities to fully utilise their talents. Positive emotions frequently increase people's effectiveness and optimism for the future, so they frequently set goals that are more ambitious than they are capable of achieving. Performance and results are inversely correlated. Positive emotions can therefore encourage employees to act more charitably and rationally, actively develop their intelligence, adopt the right attribution orientation, enhance their own work capacity, and ultimately enhance the effectiveness of teachers in the classroom.

## 3. AHP-Based Teacher Happiness Index Model

In order to explore the degree of correlation between teachers' occupational well-being and their job performance, this paper focused on exploring the happiness index under different job performance and job performance under different happiness index. The calculation of happiness index introduced the analytic hierarchy process (AHP) algorithm to establish an AHP-based teacher happiness index model.

### 3.1. Connotation of Teacher Happiness Index

1. The teacher's happiness index is not objective, but a subjective feeling [15]. Happiness is not the goal; it is just an attitude. The teacher's happiness index actually refers to the degree of satisfaction of teachers with their own occupational conditions
2. The teacher's happiness index is a kind of spiritual feeling. It is an objective judgment of life circumstances and living conditions, a value judgment of the subjective value and happiness of life, and a positive psychological experience formed based on satisfaction with living conditions
3. Teachers' happiness index is a quantitative measure of their happiness. It refers to an evaluation made by teachers on their professional status and daily life according to specific standards

### 3.2. AHP

1. Theoretical basis

AHP is an analytical method that combines qualitative and quantitative analysis and systematization and hierarchy, which can quantify and model decisions in complex systems [16]. Decision-makers need to decompose complex problems into multiple factors and multiple levels and then select the optimal solution based on the weights of these factors. This method is very effective and real-time in dealing with complex problems and has been widely used all over the world. The flow chart of AHP is shown in Figure 1.

(2) Main steps

AHP is a technique for thorough analysis and thorough decision-making. It creates a multilevel model by breaking down complex issues into various constituent parts. To assess each element's weight in its entirety and determine its relative importance, the method of double comparison is used [17]. The main steps of adopting AHP for decision-making and evaluation can typically be broken down into four stages:

- Building a hierarchically progressive model. Through the analysis of the association and affiliation between the elements in the target system, it is decomposed into different levels, thereby establishing an orderly hierarchical structure. There are usually three types of content in the established model, namely, indicators, criteria, and goals
- Building a discriminant matrix. According to the hierarchical model, the decision matrix is constructed from top to bottom. The elements of each layer are based on the elements of the adjacent previous layer, and the method used in establishing the judgment matrix is the 1-9 scaling method. Thus, a decision matrix is constructed, as shown in Table 1

(iii) Consistency check. By normalizing the largest eigenvalue in the decision matrix and the corresponding eigenvector, a single-ranked weight vector of one level is obtained. Since the conclusion of the judgment matrix is objective to a certain extent, it must be checked for consistency, and the unqualified judgment matrix must be corrected until it is consistent with the consistency standard [18]
(iv) Hierarchical total ordering. From top to bottom, comprehensive evaluation is carried out according to the level, the comprehensive weight of the index level factor and the overall goal of the whole system is obtained, and finally, the influence degree of each factor on the overall goal is determined. AHP takes priority as the evaluation index. The influence of the index ranges from 0 to 1. Under certain decision criteria, the importance of the index decreases with the increase of the index [19]. In order to determine whether the thinking is logically consistent, the overall ordering of each level must also be tested. Only the tested results can meet the requirements of analysis

The article "An Evaluation Model of Career Happiness and Job Performance of Political Teachers Based on Correlation Analysis in Positive Emotional Environment" was retracted in 2023. Reasons: signs of a paper mill; suspected computer-generated content; unreliable results or conclusions; concerns about the data.

### 3.3. Establishment and Solution of Happiness Index Model

- Teacher happiness index model

To study teachers' happiness, it is necessary to construct a scientific, reasonable, normative, and systematic evaluation index system to objectively and effectively reflect teachers' happiness, referring to the current research status of the country, synthesizing the understanding of peers, adopting the questionnaire survey method, following the basic principles of scientific validity and the combination of qualitative and quantitative, and using the AHP method to build a system model. The model established in this paper is shown in Figure 2.

(ii) Model index screening
  1. Screening step

First, a coordination group is established, and the work to each person is assigned. Secondly, the selected consultation objects are generally held by well-known experts with rich experience. Then, a consultation form is prepared to record and analyze the first round of experts. The expert consultation is carried out again. Finally, after the comparison and analysis of two rounds of expert consultation, the evaluation standard of teachers' happiness index is obtained.

(2) Screening of relevant indicators

Expert authority degree *S*_*t*_:

(1) $$\begin{array}{c} S_{t}=\frac{S_{a}+S_{b}}{2}. \end{array}$$

Weighted arithmetic mean *S*_*n*_: the higher the weight of the index element, the greater the importance, and the greater the weighted average arithmetic value, and its expression formula is shown in:

(2) $$\begin{array}{c} S_{n}=\frac{1}{i}\overset{i}{\underset{m=1}{\sum }}S_{t}S_{nm}. \end{array}$$

In the formula, *S*_*n*_ is the arithmetic weighted average of element *n*; *S*_*nm*_ is the rating value of the expert m to the element *n*; *i* is the number of experts.

Full score frequency *Q*:

(3) $$\begin{array}{c} Q=\frac{i_{n}}{i}. \end{array}$$

Grade and *T*_*n*_:

(4) $$\begin{array}{c} T_{n}=\overset{S_{n}}{\underset{n=1}{\sum }}S_{nm}. \end{array}$$

In the formula, *S*_*nm*_ is the evaluation level of the index element *m* by expert *n*.

Coefficient of variation *Vn*: another important measure of volatility is coefficient of variation, which means that different experts will have different perceptions of how much importance they place on the index. That is, the lower the coefficient of variation, the smaller the difference between experts, which means that the evaluation process is more harmonious.

Expert opinion coordination coefficient *R*: the higher the opinion coordination coefficient, the smaller the difference between the evaluations of the experts and the better the cooperation between the experts. The calculation formula is as follows:

(5) $$\begin{array}{c} R=\frac{12}{i^{2}\left(j^{3}-i\right)-i\sum_{n=1}^{i}t_{n}}\overset{i}{\underset{n=1}{\sum }}e_{n}^{2},\\ \overset{i}{\underset{n=1}{\sum }}e_{n}^{2}=\overset{i}{\underset{n=1}{\sum }}{\left(P_{n}-\bar{P}\right)}^{2}. \end{array}$$

In the formula, *e*_*n*_^2^ is the deviation of the evaluation level of the expert to the index element *n*; *i* is the total number of indicator elements; *P*_*n*_ is the evaluation level sum of index element *n*; $\bar{P}$ is the mean value of the sum of the evaluation grades of all the index elements.

(6) $$\begin{array}{c} d_{i}=\overset{L}{\underset{l=1}{\sum }}\left(d_{l}^{3}-d_{l}\right). \end{array}$$

In the formula, *L* is the same number of groups in the expert evaluation value; *d*_*l*_ is the number of identical levels in the group.

(iii) Judgment matrix is constructed, and eigenvectors are calculated

In the AHP method, there are two calculation methods for calculating the maximum eigenvalue and eigenvector of the decision matrix, namely, the summation method and the root-finding method. Here, the root-finding method is used to calculate. The process is as follows:

1. After multiplying the elements of each row, the root of the *i* power is found:

(7) $$\begin{array}{c} \bar{\alpha_{n}}=\sqrt[{i}]{\overset{i}{\underset{m=1}{\prod }}a_{nm}}. \end{array}$$

In the formula: *n* = 1, 2, 3, ⋯, *i*.

(2) After normalization, it is:

(8) $$\begin{array}{c} \alpha_{n}=\frac{\bar{\alpha_{n}}}{\sum_{n=1}^{i}\bar{\alpha_{n}}},\\ A={\left(\alpha_{1},\alpha_{2},\cdots ,\alpha_{i}\right)}^{T} \end{array}$$

(3) The lines are added to get ${\bar{R}}_{n}$:

(9) $$\begin{array}{c} {\bar{R}}_{n}=\overset{i}{\underset{n=1}{\sum }}a_{nm} \end{array}$$

(4) The rows are normalized to get the weight coefficient *R*_*n*_:

(10) $$\begin{array}{c} R_{n}=\frac{{\bar{R}}_{n}}{\sum_{n=1}^{i}{\bar{R}}_{n}} \end{array}$$

(5) Judgment test for the consistency of the matrix, assuming that *α*_max_ is the maximum eigenvalue of the judgment matrix, and the judgment calculation formula of the maximum eigenroot is:

(11) $$\begin{array}{c} \alpha_{\max}=\frac{1}{i}\underset{n}{\sum }\frac{{\left(BR\right)}_{n}}{R_{n}},\\ \text{CI}=\frac{\alpha_{\max}-i}{i-1} \end{array}$$

(iv) Vector consistency test

When *i* = 4, the index parameters given in Table 2 is referred to obtain the consistent average random index RI. According to the obtained value, the consistency ratio can be calculated:

(12) $$\begin{array}{c} \text{CR}=\frac{\text{CI}}{\text{RI}}. \end{array}$$

In the case of CR > 0.1, the consistency of the matrix is unsatisfactory, which indicates that the weights of the first-level indicators are not reliable. On the contrary, the results obtained by the model are consistent. That is, the weights of the first-level indicators are effective and credible, and finally, the weights of the first-level indicators can be determined [20], as shown in Table 2.

The article "An Evaluation Model of Career Happiness and Job Performance of Political Teachers Based on Correlation Analysis in Positive Emotional Environment" was retracted in 2023. Reasons: signs of a paper mill; suspected computer-generated content; unreliable results or conclusions; concerns about the data.

## 4. Results of Happiness Index

In this paper, 200 political teachers from 20 different schools were investigated by means of a questionnaire survey. The distribution of the selected experimental survey objects is shown in Table 3.

Job performance surveys are conducted, and political teachers of different school levels and different teaching ages are interviewed; the survey results and organize data are collected, and statistics on the scores of four factors of political teachers' occupational well-being is made. The four well-being factors are psychological well-being, emotional well-being, social well-being, and cognitive well-being. The scores of different well-being factors are shown in Figure 3.

Figure 3 shows that, firstly, if the factors of different political teachers' occupational well-being are sorted according to the mean score, they are emotion, cognition, society, and psychology from small to large. Second, the difference between the different factors of political teachers' occupational well-being is the largest at 27 and the smallest at 10.1. Third, the factor that achieves the maximum score is cognitive well-being, with a maximum value of 29, while the factor that achieves the minimum score is emotional well-being, with a minimum value of only 2.

The professional well-being of political teachers can also be divided into three factors, namely, work dedication, human-machine promotion, and task performance. The scores of these three job performance factors of teachers are summarized and counted, and the results are shown in Figure 4.

Figure 4 shows that, first, if the different factors of political teachers' work performance are sorted according to the average score, they are work dedication, interpersonal promotion, and task performance from small to large. Second, the difference between the scores of different factors of political teachers' work performance is 79 at the maximum and 22 at the minimum. Third, the job performance factor that achieves the maximum score is task performance, and the maximum value is reached, while the job performance factor that achieves the minimum score is job dedication, and the minimum value is only 12.

The scores of different job performance factors are integrated to obtain the total score of job performance. This paper conducted a classified survey on political teachers of different teaching ages and political teachers in schools of different levels to ensure the universality of the experimental results and calculated the total score of work performance and its average value. The survey results are shown in Figure 5.

The article "An Evaluation Model of Career Happiness and Job Performance of Political Teachers Based on Correlation Analysis in Positive Emotional Environment" was retracted in 2023. Reasons: signs of a paper mill; suspected computer-generated content; unreliable results or conclusions; concerns about the data.

As can be seen from Figure 5, the average total score of political teachers with more than 6 years of teaching experience exceeded 90%. There is little difference in job performance. For school teachers of different levels, the job performance of university political teachers was often much lower than that of middle school teachers, and the average job performance total score was lower than 70%. The reason is that the discipline of university classrooms is lower than that of middle schools, and students have a strong sense of autonomy, resulting in relatively poor teaching effects.

Then, statistical analysis was carried out on the happiness of these survey subjects, and the scores of different occupational happiness factors were integrated to obtain the total score of happiness, as shown in Figure 6.

Figure 6 shows that, on average, female political educators are happier than their male counterparts, suggesting that women educators are more likely to find fulfilment in their careers as educators. Greater happiness is also predicted for teachers who are older in the classroom. It is generally accepted that as teachers get older, they are happier in their jobs. This is frequently due to the fact that teachers who are older in age when they begin teaching typically have higher pay and less stress at work. A promotion is not required of them because they already hold higher professional titles. College instructors typically report a higher sense of well-being than middle school instructors, who report a relatively low sense of well-being.

Analyzing correlations between various aspects of job performance and the professional well-being of political teachers using experimental data is done.  Table 4 presents the analysis' findings.

It can be seen from Table 4: first, the correlation of the total score between the surveyed political teachers' occupational well-being and job performance is very obvious, among them, *r* = 0.799, *P* < 0.01. Second, there is a significant relationship between the total score of job performance and the four factors of teachers' professional well-being, and the average correlation coefficient *r* reached 0.65. Third, there is a significant relationship between the total score of political teachers' occupational well-being and the three factors of job performance, with an average correlation coefficient of 0.73. Fourth, except for the low correlation between emotional well-being and interpersonal promotion, the correlations between other happiness factors and job performance factors are relatively obvious.

## 5. Conclusion

In this paper, 200 selected political teachers were interviewed and investigated in the form of questionnaires, and their job performance and occupational well-being were descriptively analyzed and compared in the form of data scores. The experimental results showed that (1) political teachers have better job happiness, at the middle and upper level, political teachers with more than 6 years have the highest job happiness, and political teachers with less than 1 year have the lowest happiness. Political teachers have good job performance and are the best performers between 6 and 9 years, and new class teachers have the lowest job performance. (2) With the higher professional well-being of political teachers, their daily work performance will also improve, and their psychological well-being and cognitive well-being have a more obvious impact on their work performance. However, there are also some defects in this article, for example, when analyzing the work performance of political teachers, it does not take into account the educational background of teachers, resulting in the lack of high generality of the experimental results. Therefore, it needs to be developed and improved in future research.

The article "An Evaluation Model of Career Happiness and Job Performance of Political Teachers Based on Correlation Analysis in Positive Emotional Environment" was retracted in 2023. Reasons: signs of a paper mill; suspected computer-generated content; unreliable results or conclusions; concerns about the data.

## Figures and Tables

**Figure 1:** AHP flow chart

**Figure 2:** Teacher happiness index model.

**Figure 3:** Political teachers' occupational well-being factor scores.

**Figure 4:** Political teachers' job performance factor scores.

**Figure 5:** Average total score for job performance.

**Figure 6:** Average total score of teachers' occupational well-being.

**Table 1:** Scale meaning.

Scaling	Definition	Meaning
1	Equal importance	Two elements are equally important to a criterion
3	Slightly important	Two elements are slightly more important than the latter for a criterion
5	Obviously important	Two elements for a criterion, the former is obviously more important than the latter
7	Strongly important	Two elements are strongly important to a criterion, the former is more important than the latter
9	Extremely important	Two elements are extremely important to a criterion, the former is more important than the latter
2, 4, 6, 8	Neighbor scale median	A scale that represents a compromise between two adjacent scales

**Table 2:** Average random consistency index.

Order	1	2	3	4
RI	0	0	0.58	0.9
Order	5	6	7	8
RI	1.12	1.24	1.32	1.41

**Table 3:** Detailed distribution of teachers.

	0~1 year	2~5 years	6~9 years	10+ years	Total
Primary school teachers	18	27	24	15	84
Middle school teacher	15	20	17	11	63
University teacher	13	20	11	9	53
Total	46	67	52	35	200

**Table 4:** Correlation between career well-being and job performance of political teachers.

Occupational well-being factor	Task performance	Interpersonal promotion	Work dedication	Overall job performance score
Psychological well-being	0.628	0.655	0.576	0.698
Emotional well-being	0.628	0.077	0.543	0.477
Social well-being	0.605	0.552	0.651	0.682
Cognitive well-being	0.622	0.543	0.671	0.693
Total occupational happiness score	0.774	0.570	0.761	0.799

The article "An Evaluation Model of Career Happiness and Job Performance of Political Teachers Based on Correlation Analysis in Positive Emotional Environment" was retracted in 2023. Reasons: signs of a paper mill; suspected computer-generated content; unreliable results or conclusions; concerns about the data.

## Data Availability

The data used to support the findings of this study are available from the corresponding author upon request.
